# Determinants of the Severity of Contract Enforcement in Chinese PPP Projects: From Public Sector's Perspective

**DOI:** 10.1155/2022/5149478

**Published:** 2022-09-02

**Authors:** Xiaodan Zheng, Shaojie Wang, Yuchen Yang

**Affiliations:** Department of Construction Management, College of Civil Engineering, Nanjing Forestry University, Nanjing 210037, China

## Abstract

In PPP projects, the enforcement of concession contract is of much importance. Thus, this study analyzed the severity of contract enforcement after private sectors violate concession contracts in Chinese PPP projects from the perspective of public sectors. Through 39 in-depth interviews with those working in public sectors under Chinese PPP projects, there were four determinants identified for the severity of contract enforcement in public sectors: the consequence of contract violations, the intention of contract violations, private sectors' remedies, and private sectors' prior performance. Furthermore, this study analyzed the intrinsic relationship between the four determinants with trust foundation, destruction, and repair. The findings of this study extend the existing theory on the severity of contract enforcement. For those managers working in public sectors, the findings of this study can help improve their flexibility in contract enforcement, thus contributing to the success of PPP projects.

## 1. Introduction

To relieve financial pressures on governments and give full play to the market efficiency, an increasing number of countries use PPP (Public Private Partnership) to develop infrastructure projects. According to the Private Participation in Infrastructure (PPI) Project Database, the private investment commitments in low- and middle-income countries amounted to US$45.7 billion in 2020 across 252 projects, and then to US$76.2 billion in 2021 across 240 projects [1].

In PPP projects, public and private sectors sign concession contracts to establish a long contractual relationship. According to China PPP Center, many of the concession contracts signed in China can last 20 to 30 years [2]. As for concession contracts, the existing studies focus mainly on contract design [3–5] and contract renegotiation [6–8]. However, there is little attention paid to the enforcement of concession contracts. In fact, it is usually assumed in the existing studies that concession contract enforcement is severe. For example, Klijn and Koppenjan [9] argued that there was a need to impose sanctions to enforce concession contracts in PPP projects. Yue and Lin [10] suggested that when private sectors provided low-quality services in PPP projects, they should be subjected to punishment according to the concession contracts. However, when PPP projects are undertaken in China, it is common that when there are contract violations in private sectors, public sectors do not strictly comply with the breach clauses to severely punish private sectors. Why do public sectors reduce the severity of contract enforcement in China? The existing studies fail to answer this question.

Given a long-term contractual relationship, it is common for contract violations to occur. Since private sectors are profit-driven, it is likely for them to engage in opportunistic behaviors and defaults for the maximum benefits of their own [11, 12]. Thus, it is necessary to analyze why public sectors in Chinese PPP projects have different severities of contract enforcement, which is conducive to better understanding the enforcement of concession contract in China.

Therefore, this study identifies determinants of the severity of contract enforcement after private sectors violate concession contracts in Chinese PPP projects from the perspective of public sectors. The findings of this study are expected to help public sectors take more flexible disciplinary actions against those private sectors with contract violations, so as to improve the efficiency of concession contract fulfillment and ensure the success of PPP projects.

## 2. Literature Review

### 2.1. The Severity of Contract Enforcement

The severity of contract enforcement is defined as “the severity of a principal's (i.e., the party offering the contract) disciplinary response to an agent's (i.e., the party accepting the contract) violation of a contractual obligation” [13, 14]. In a certain PPP concession contract, the principal is the public sector (i.e., the public sector offering the concession contract) and the agent is the private sector (i.e., the private sector accepting the concession contract). Thus, for the PPP concession contract, the severity of contract enforcement refers to the severity of disciplinary response from a public sector to the violation of the contractual obligation by a private sector.

The severity of contract enforcement is a continuous variable. It ranges from lenient actions, such as ignoring the violation entirely or making only mild attempts, to tough and punitive actions, such as strict cease-and-desist orders or termination proceedings [13]. It has been found out in prior research that the severity of contract enforcement can affect the satisfaction with problem resolution [15], opportunism [16], cooperation [17], relationship performance [18], and project performance [19].

### 2.2. Antecedents of the Severity of Contract Enforcement

Given a significant role played by the severity of contract enforcement in the stage of contract performance, scholars also analyze the antecedents of the severity of contract enforcement. First of all, the severity of contract enforcement can be affected by the characteristics of the contract itself. For example, Faems et al. [20] revealed that a rigid contract enforcement would result from the narrow contractual interface structure of research and development projects, while a flexible contract enforcement would result from the broad contractual interface structure of them. With regard to channel management, contract ambiguity can reduce the severity of contract enforcement [13].

Secondly, the severity of contract enforcement can be affected by transactional attributes. For example, in the channel relationships, the principal is expected to respond with a relatively severe enforcement when transaction-specific investments are high, or when the contractual obligations of each other are highly interdependent [13]. Given a high likelihood of future continued trading, the severity of contract enforcement can be mitigated for construction projects [21].

Thirdly, the relationship between two contracting parties can affect the severity of contract enforcement. For example, the prior ties in construction projects play a role in reducing the severity of contract enforcement [21]. And trust and relationalism between two contracting parties are negatively associated with the severity of contract enforcement [13, 14, 19].

Finally, external environment can make a difference to the severity of contract enforcement. For example, according to Antia and Frazier [13], the rapid change of external environment increased the severity of contract enforcement in the channel relationships because the principal intended to maintain control. At the same time, culture also affects the severity of contract enforcement. There is a variation in the severity of business contract enforcement between Eastern and Western countries [22, 23].

### 2.3. Concession Contracts in PPP Projects

Under PPP projects, concession contracts define the rights and obligations of both public and private sectors, which guide them to cooperate with each other in undertaking the projects [24]. Since concession contracts are essential for PPP projects, scholars attach much significance to the study of concession contracts. Up to now, there have been many scholars exploring how to better design concession contracts. They researched plenty of important issues in concession contracts, such as determining the optimal concession period [25, 26], capital structure [27], contract change mechanism [5], contract content flexibility [28], and contract completeness [24].

In addition, the long project cycle and considerable uncertainty of PPP projects may require that adjustment is made to the original concession contract during the implementation of PPP projects [29]. Therefore, scholars have also studied concession contract renegotiations in the context of PPP projects. For example, Cruz et al. [6] identified the incentives of concession contract renegotiations. Khallaf et al. [30] analyzed the decision-making of renegotiations in PPP projects. Lv et al. [8] explored the evolvement of concession renegotiation behaviours. Xiong et al. [31] investigated how public values were influenced by concession contract renegotiations.

### 2.4. Research Gap

According to literature review, it can be found that previous studies recognized the role of the severity of contract enforcement and discussed the antecedents of the severity of contract enforcement. However, these studies did not focus on the severity of contract enforcement in the context of PPP projects. They did not discuss why the severity of contract enforcement varied in public sectors after concession contracts were violated by private sectors. In fact, different research situations can have a significant impact on the research results [32]. PPP projects are characterized by heavy investment, long project cycle, strong asset specificity, and high lock-in degree [33–35]. In addition, although the concession contract of the PPP project is signed between the public and private sectors, the PPP project can have an immediate effect on the public interest, which in turn can influence the decision-making of the public sector [36]. Due to these complex characteristics of PPP projects, the determinants of the severity of concession contract enforcement in public sectors may be inconsistent with previous research results. Therefore, it is necessary to explore the determinants for the severity of contract enforcement in public sectors after concession contracts are violated by private sectors under PPP projects. In addition, culture can also affect the severity of contract enforcement [22, 23]. The focus of this study is the Chinese PPP projects.

## 3. Methodology

### 3.1. Research Design

This study is an explorative study to identify the determinants for the severity of contract enforcement in public sectors after the violation of concession contracts in private sectors under Chinese PPP projects. The in-depth interview research method is considered appropriate for this study, because an in-depth interview supports researchers in collecting plenty of data on the research questions. On this basis, the answers to the research questions can be induced and found when the relevant literature is limited [37].

### 3.2. Data Collection

In this study, semi-structured interviews were conducted to collect data. Semi-structured interviews are positioned between unstructured interviews and structured interviews. Compared with unstructured interviews, semi-structured interviews are more effective in guiding informants to express their personal view on the selected topics. In comparison with structured interviews, most of the questions in semi-structured interviews are open-ended ones, which allow the informants sufficient freedom to share their own viewpoints. Also, in semi-structured interviews, the interviewers can raise additional questions beyond the interview protocols according to the response from informants, so as to find out about other interesting research phenomena [38].

In this study, the potential informants were recruited from a PPP workshop held in Fuzhou, China, in 2021. Most of the participants in the PPP workshop were from public sectors, private sectors, or academia. This study focused on the severity of contract enforcement in public sectors under Chinese PPP projects. For this reason, the participants working in public sectors under Chinese PPP projects were selected to comprise an alternative name list. There were 48 people on this list. Hard-copy interview invitation letters were sent to these 48 people, introducing the purpose, main content, and process of the interview. Subsequently, 39 people agreed to take the interview. Therefore, these 39 people became informants to share their experience of concession contract enforcement. As indicated by Yin (2003), interviews can be terminated in case of data saturation which is the time point when researchers are unable to collect more new information from additional informants. In this study, data saturation was reached after 26 interviews were completed. Afterwards, another 13 interviews were conducted to ensure that no new information can be gathered. The 39 informants included 33 males and 6 females. Most of the informants had spent more than three years working in public sectors under Chinese PPP projects. The types of PPP projects that they had worked on included sewage treatment, waste disposal, transportation, government-subsidized housing, ecological and environmental conservation, schools, the sponge city, and so on.

Each interview was conducted one-on-one and face-to-face, with the native language of informants used. During the interview process, the interviewer raised questions mainly according to the interview protocol. In some cases, additional questions were raised according to the response of the informants.  Table 1 lists the questions shown in the interview protocol. The informants were encouraged to elaborate upon their viewpoints by using specific events and examples rather than abstract concepts. On average, each interview lasted 50 minutes. All of the interviews were tape recorded, transcribed, and returned to the informants in the form of feedback.

### 3.3. Data Analysis

For the interview data analysis, a content analysis was conducted in this study by following the procedure specified by Wang et al. [1] and Zheng et al. [39]. First of all, each sentence in each individual transcript was reviewed and understood. Secondly, for each individual transcript, the informant's words describing the contract violation in one private sector and the disciplinary response from the public sector were extracted and coded into an item. Thirdly, for each item, the determinants of the severity of contract enforcement in public sectors were summarized. Fourthly, all the determinants from different items were compared, and the similar determinants from different items were combined to obtain new determinants. Each new determinant was named and given a general description and interpretation according to its features. In addition, only those determinants as mentioned by more than one informant were used, so as to prevent informant bias. If a determinant was mentioned by only one informant, it was removed. Finally, to ensure research validity, the results were sent to all informants via e-mail after the completion of data analysis. Given the feedback collected from all informants, the results were modified accordingly.

## 4. Determinants of the Severity of Contract Enforcement in PPP Projects

According to the in-depth interviews, there were four determinants identified for the severity of contract enforcement in public sectors after concession contracts were violated by private sectors in Chinese PPP projects: the consequence of contract violations, the intention of contract violations, private sectors' remedies, and private sectors' prior performance.

### 4.1. The Consequence of Contract Violations

According to the informants, to determine the severity of contract enforcement, the first thing to do was to estimate whether the breach of concession contract by a private sector had caused serious adverse consequences to the public sector or the public interest. If the contract violations caused substantial losses to public sectors or public interests, severe contract enforcement can be applied by public sectors to punish private sectors. As explained by the informants, severe contract enforcement can make up for losses. Moreover, severe contract enforcement can mitigate the potential risks of future violations by warning and deterring private sectors. Furthermore, if the public interests were severely damaged by contract violations, it was likely to cause public discontent. In this case, it was also necessary for public sectors to punish private sectors severely, so as to appease public discontent.

On the contrary, if the contract violations by private sectors caused slight losses or no loss to public sectors or public interests, lenient contract enforcement may be applied by public sectors, such as persuasion. As further explained by the informants, the disciplinary action here was not purposed to compensate for the loss, but to persuade private sectors to behave better in the future. Also, the very long project cycle of PPP projects required a long-term collaboration between public and private sectors. If public sectors punished private sectors severely for a minor mistake, it may seem too impersonal, which may make private sectors hostile, thus leading to a long-term bad relationship.

### 4.2. The Intention of Contract Violations

As stated by the informants, the incentive of private sectors to default was also important in determining the severity of contract enforcement, whether it was intentional, negligent, incompetent, or opportunistic. If it was found out by public sectors that the concession contract violations by private sectors were intentional and opportunistic, private sectors were considered as dishonest and unreliable. Therefore, public sectors must rely on the coercive deterrence of contracts to govern a bilateral relationship and have severe contract enforcement. Due to the harsh penalties imposed by public sectors, private sectors understood that opportunistic behaviors can lead to serious losses for itself. In addition, the losses must outweigh the gains from opportunism. Therefore, after weighing the gains and losses of opportunistic behaviors, private sectors would give up opportunistic behaviors in the future. In contrast, if leniency was given by public sectors to private sectors at this time, not only would it be difficult to deter private sectors, private sectors would also be encouraged to “push its luck” (i.e., to continue contract violations and opportunistic behaviors in the future).

However, if the concession contract violations by private sectors were found to be unintentional, public sectors may be willing to forgive private sectors, with no severe contract enforcement involved. In this case, the leniency of public sectors led private sectors to believe that public sectors were understanding and reasonable. It may win the private sector's gratitude and reciprocity, which can further strengthen the emotional ties between the two sides and foster a long-term partnership.

### 4.3. Private Sectors' Remedies

As mentioned by the informants, if private sectors took remedies after a default, remedies were another significant factor to determine the severity of contract enforcement. If appropriate remedial measures were adopted by private sectors, it demonstrated that private sectors regretted violations, genuinely intended to correct it, and expected to continue cooperative relationship. These are effective in increasing the willingness and confidence of public sectors to continue the partnership. Thus, public sectors can reduce the severity of contract enforcement to maintain the partnership. In addition, when the contract violations by private sectors damaged public interests and triggered public opposition, if private sectors can take appropriate remedies to appease the public and eliminate the public opposition, it can alleviate the pressure exerted on public sectors in terms of public opinion, so as to change the negative impression left by private sectors on public sectors. It may also reduce the severity of contract enforcement by public sectors.

On the contrary, if private sectors showed perfunctory attitudes in taking corrective actions, it indicated that private sectors did not realize the seriousness of the problems. Then, it was necessary for public sectors to increase the severity of contract enforcement, thus giving private sectors adequate punishment and warning. In addition, public sectors may be further enraged by the perfunctory attitudes and remedies, which would make the punishment severer for private sectors.

### 4.4. Private Sectors' Prior Performance

According the informants, to determine the severity of contract enforcement, the prior performance of private sectors would be also taken into account to some extent. If private sectors performed well and had no default in the past, and this was the first-time default, it indicated that the competence and cooperative intentions of private sectors were qualified. This default may be simply an accident and the risk of recurrence was low. Thus, public sectors may adopt low severity of contract enforcement and even help private sectors jointly solve problems from the perspective of solidarity for maintaining long-term partnerships. The informants added that, in this case, leniency may make private sectors perceive the goodwill of public sectors, thus boosting the confidence of private sectors in the partnership. As a result, private sectors may reciprocate with better performance in the future.

On the other hand, if private sectors had a poor track record and had defaulted frequently in the past, it signaled that private sectors lacked the competence and integrity required to fulfill their contractual obligations. Then, only by imposing severe punishment on private sectors can they be made to realize the scale of problems and seek to make improvements. The informants also mentioned that frequent defaults would make public sectors loathe private sectors, so that private sectors should be subjected to tough punishment from an emotional perspective. The informants added that, if private sectors defaulted repeatedly and there was no good turnaround, public sectors may choose to terminate concession contracts early and find other partners. This was because public sectors must stop making loss possibly soon. Moreover, if private sectors repeatedly defaulted and jeopardized public interests, it would be very likely to cause public opposition. If the public pressurized governments into ending private participation, public sectors would have to terminate concession contracts early.

Table 2 shows these four determinants. In addition, all of the informants stressed that there was no single factor that determined the severity of concession contract enforcement in PPP projects but a combination of several factors. For example, even if the contract violations of private sectors were not severe, but private sectors had deliberately defaulted many times in the past, public sectors can enforce contracts more rigorously. This was because multiple deliberate defaults suggested that private sectors were opportunistic. Thus, it was necessary to curb the opportunistic tendencies of private sectors by imposing strict penalties, whereas weak penalties played no role in deterring opportunism. On the contrary, if the default of private sectors caused serious consequences, but active remedial actions were taken by private sectors to minimize the losses suffered by public sectors, the severity of contract enforcement would be reduced by public sectors as appropriate.

## 5. Discussion

In this study, it was discovered that for the concession contracts under Chinese PPP projects, the prior performance of private sectors would affect the severity of contract enforcement to some extent. Previous studies on the severity of contract enforcement had similar findings, suggesting that prior collaboration was negatively associated with severe contract enforcement [21]. The commonality between past performance and past collaboration lies in a direct impact on the trust foundation. The improvement of past performance or past collaboration can reinforce the trust foundation [40–42]. For example, Smyth and Edkins [43] and Zou et al. [44] demonstrated that if private sectors had good performance in PPP projects, public sectors could build the high level of trust in them. Conversely, if the performance of private sectors failed to satisfy public sectors, a low level of trust would be shown by public sectors in private sectors. This suggests that the prior performance of private sectors can affect the severity of contract enforcement by influencing the foundation of the trust placed by public sectors in private sectors. When the trust foundation is strong, the contract enforcement becomes less strict [19].

Both the consequence and intention of contract violations are part of the characteristics of contract violations. That is to say, the severity of contract enforcement in Chinese PPP projects can be affected by the characteristics of private sectors violating concession contracts. However, previous studies paid little attention to the impact of contract breach itself on the severity of contract enforcement. But past studies about trust violations had found similar results. It was discovered that the different characteristics of trust violations affected the extent to which trust was undermined [45]. When the consequence of trust breach was serious or the intention of it was malicious, trust would be eroded to a significant extent [46–49]. This was basically consistent with the findings of this study. It was found out in this study that the contract enforcement by public sectors would be severe when the consequence of the private sector's contract breach was serious or the intention of it was opportunistic. This shows that contract violations and the severity of contract enforcement are closely related to trust violations. A contract violation can erode the trust of the violated party in the violating party [50]. The severer the breach of contracts, the more significant the breach of trust. When the violated party's trust is seriously broken, the violated party will be enraged. In response, they will impose severe penalties on defaulters (i.e., high severity of contract enforcement). On the contrary, when the breach of the contract is relatively minor, the breach of trust is also relatively insignificant. In this circumstance, the violated party will have relatively mild punishment, rather than severely punishing defaulters (i.e., low severity of contract enforcement).

It was also revealed in this study that the remedies adopted by private sectors after concession contract violations would make difference to the severity of contract enforcement in Chinese PPP projects. When private sectors adopted positive remedies after defaults, the severity of contract enforcement would be reduced. This finding is also what has not been addressed by the past studies on the severity of contract enforcement. However, this finding is closely related to trust repair. According to the research of trust repair, trust can be repaired by adopting appropriate trust repair strategies [39, 51]. For example, substantive strategies, such as financial compensation, are more effective in repairing trust than simply making verbal apologies or explanations [52, 53]. It demonstrates that the appropriate remedies can be relied on to repair the trust destroyed by defaults. When trust is better restored, the severity of contract enforcement is reduced.

Therefore, different from previous studies, this study linked the severity of contract enforcement with PPP concession contracts. The findings of this study not only supplemented the lack of consideration given to the impact of characteristics of contract violations and remedies on the severity of contract enforcement but also linked contract violations and the severity of contract enforcement with trust violations and repair. It was found out that trust may be undermined by contract violations, and the degree to which trust was eroded can affect the severity of contract enforcement. Meanwhile, the remedies taken after defaults can help repair the damaged trust to a certain extent, and the degree of trust being repaired would also affect the severity of contract enforcement. In addition, based on previous studies, it was also found in this study that trust basis also affected the severity of contract enforcement to some extent. In the case of a strong trust base, the severity of contract enforcement was reduced as appropriate. Therefore, this study revealed that the essence of trust influencing the severity of contract enforcement was determined by trust foundation, destruction, and repair in combination. Although previous studies also explored the impact of trust on the severity of contract enforcement, proposing a negative correlation between the trust level and the severity of contract enforcement [14, 19, 21], there was still no in-depth analysis as to the nature of the impact. Thus, the findings of this study are expected to further expand the research perspective on the severity of contract enforcement.

In addition, Chinese culture can also make an impact because this study discussed the severity of contract enforcement for concession contracts in Chinese PPP projects. As for the relationship between law, reasons, and emotion, the Western culture attaches more importance to law than to reasons and emotion. Since contracts are regarded as the private laws between two contracting parties, the Western culture tends to strictly comply with contracts in punishing defaulters. However, in the Confucian culture of China, people attach more significance to emotion and reasons than to law [54]. If it is considered reasonable, it can be lenient, which explains why the PPP projects in China often fail to severely punish defaulters in accordance with the concession contracts. Just as in the interviews, when the interviewees explained why the severity of contract enforcement was reduced, they repeatedly mentioned such words as “relationship,” “emotion,” “understanding and reasonable,” and “excusable.” It is because of emotion and reasons that the severity of contract enforcement for concession contracts in Chinese PPP projects is affected by prior performance and the intention of contract violations. When prior performance is good, merits offset faults for dealing with a default. When the breach is extenuating, leniency is chosen. Moreover, the Confucian culture also values the correction and shows tolerance to those who can correct their mistakes. Under the influence of this idea, the remedies taken after breach of concession contracts also have a significant impact on the severity of contract enforcement in Chinese PPP projects. Finally, the Confucian culture also places emphasis on moderation, which makes people incline to leave some leeway for punishing defaulters, rather than resorting to extreme punishments. Therefore, the findings of this study may be more suitable as reference for the PPP projects undertaken in those Asian countries influenced by the Confucian culture. For Western countries, the results of this study could allow Western companies to better understand the contract enforcement in Chinese public sectors, which is conducive for their participation in Chinese PPP projects.

## 6. Conclusion

This study explored the severity of contract enforcement by public sectors after concession contracts were violated by private sectors in Chinese PPP projects. Through 39 in-depth interviews, there were four determinants of the severity of contract enforcement identified, including the consequence of contract violations, the intention of contract violations, the remedies taken by private sectors, and the prior performance of private sectors, respectively. Besides, further analysis was conducted as to the intrinsic relationships between the four determinants with trust foundation, destruction, and repair. Therefore, this study extends the existing theory on the severity of contract enforcement. In practice, the findings of this study are expected to support public sectors in adopting contract enforcement in a more flexible way according to the characteristics of contract violations, and the remedies and prior performance of private sectors, so as to prevent concession contract violations from recurrence and maintain a long-term partnership. At the same time, the findings of this study can also guide the violating private sectors to make up for their violations as much as possible for diminishing the severity of contract enforcement.

There are some limitations and future research topics. Firstly, this study focused on PPP projects in China, with all the interviewees coming from China. However, the culture can have an influence. Thus, future research can be conducted to further explore the determinants of the severity of contract enforcement in PPP projects in Western countries and compare the differences between Eastern and Western cultures. Secondly, it was found in this study that the severity of contract enforcement was not determined by a single factor, but by multiple factors. Therefore, future research can quantify the influence paths of multiple determinants on the severity of contract enforcement [55].

## Figures and Tables

**Table 1:** Questions in the interview protocol.

	Questions
First part	How long have you worked in public sectors in PPP projects?
	What kind of PPP projects are you engaged in?
	What are your position and job responsibilities in the PPP projects?
Second part	Have your sector ever experienced private sector's contract violations during PPP projects? Could you please give me some examples?
	If yes, how did your sector respond to the private sector? Did your sector strictly comply with breach clauses to punish the private sector?
	Why did your sector have the response to the private sector's violation?

**Table 2:** The determinants of the severity of contract enforcement in PPP projects.

Determinants	Effects
The consequence of contract violations	If the concession contract violations by private sectors caused serious losses to public sectors or public interests, severe contract enforcement can be applied by public sectors to punish private sectors.
	If the concession contract violations by private sectors caused slight losses or no loss to public sectors or public interests, public sectors may apply lenient contract enforcement.
The intention of contract violations	If it was found out by public sectors that the concession contract violations by private sectors were intentional and opportunistic, public sectors must adopt severe contract enforcement.
	If the concession contract violations by private sectors were unintentional, public sectors may not adopt severe contract enforcement.
Private sectors' remedies	If private sectors adopted appropriate remedial measures, public sectors can reduce the severity of contract enforcement.
	If the corrective attitudes and measures of private sectors were perfunctory, public sectors should increase the severity of contract enforcement.
Private sectors' prior performance	If private sectors performed well and had no default in the past, public sectors may adopt low severity of contract enforcement and even support private sectors in solving problems.
	If private sectors had a poor track record and had defaulted frequently in the past, public sectors can severely punish private sectors, and even consider terminating concession contracts early.

## Data Availability

The interview data used to support the findings of this study are available from the corresponding author upon request.
